# Diagnosis of Chronic Kidney Disease by Three-Dimensional Contrast-Enhanced Ultrasound Combined with Augmented Reality Medical Technology

This article has been retracted.

**DOI:** 10.1155/2021/5542822

**Published:** 2021-03-16

**Authors:** Yan Zhuang, Juanjuan Sun, Jiaqiang Liu

**Affiliations:** ^1^Department of Nephrology, Linyi Central Hospital, Linyi 276400, Shandong, China; ^2^Hemodialysis of Linyi Central Hospital, Linyi 276400, Shandong, China

## Abstract

Chronic kidney disease is a worldwide clinical and public health problem. As a risk factor for cardiovascular and cerebrovascular diseases, the disease has gradually become one of the causes of morbidity and death. As a routine method of screening for kidney disease, ultrasound is very important in improving the rate of early detection and accuracy of chronic kidney disease. This article explores the value of applying 3D ultrasound in conjunction with augmented reality medical technology in chronic kidney disease, observing changes in kidney tumor at different stages with percutaneous 3D ultrasound in patients with chronic kidney disease. Volunteers with chronic kidney disease were selected for this experiment. Among them, 160 males and 140 females were diagnosed as chronic kidney disease by clinical or renal pathological biopsy, and they all met the K/DOQI diagnostic criteria for chronic kidney disease. The selected subjects met the criteria and were divided into 5 groups, each with 60 patients, to explore the correlation of properties such as three-dimensional ultrasound kidney volume in different stages of chronic kidney disease. Experiments have shown that, with the increase in the stages of chronic kidney disease, the elasticity and volume of the renal parenchyma decrease, and the resistance index of the renal artery becomes larger, *P* < 0.05; the difference is statistically significant, indicating that the elasticity of the renal parenchyma is associated with chronic kidney disease. The stage is negatively correlated, and the resistance index of the renal artery is positively correlated with the stage of chronic kidney disease. That is, as the stage of chronic kidney disease increases, the three-dimensional volume of the kidney shows a decreasing trend and the resistance index of the renal artery shows an increasing trend. Speed shows a declining trend and there is some correlation between the three.

## 1. Introduction

The traditional process of diagnosing a disease is mainly based on the patient's subjective feelings and oral description of the physical condition. The doctor combines the patient's own professional knowledge and experience, uses the patient's response to judge the disease, and determines the pathological condition through certain examinations to help the treatment process. This medical diagnosis system combines the subjectivity of patients and doctors. In addition, different patients have different manifestations of disease. For patients with weaker susceptibility, the manifestations of the disease may be different. In this case, it can lead to diagnostic errors and has major limitations. Therefore, in the method of acquiring medical knowledge, various factors must be considered as a whole in order to reduce the subjective involvement of physicians and patients. As a routine test for kidney disease, ultrasound is needed to improve the early detection rate and accuracy of chronic kidney disease [1].

There have been many research results in 3D ultrasound technology and augmented reality technology abroad. The research of 3D ultrasound technology in medical disease prediction mainly uses actual medical data to construct predictive models and uses actual applications or medical data for testing and models. The Schalk study found that, in terms of kidney volume measurement, three-dimensional ultrasound is better than two-dimensional ultrasound in terms of reproducibility, and three-dimensional ultrasound can more intuitively observe the shape and structure of the kidney [2]. Shimada used a low-MI continuous imaging method to obtain appropriate tissue suppression but at the same time maintain sufficient penetrating power, and placed the focus on the deep side of the observation target [3]. Green proposed that the kidney length includes renal sinus fat, which cannot truly reflect the size of functional renal tissue. Since renal parenchyma does not contain renal sinus fat, the measurement of its thickness can well reflect the size of functional renal tissue [4].

In recent years, there have been more and more researches on 3D ultrasound technology and augmented reality technology in China. With the improvement of science and medical technology [5], the research on 3D ultrasound technology and augmented reality technology has become more and more mature. The reproducibility of measuring kidney volume is better than that of two-dimensional, and it is gradually used in clinical evaluation of kidney disease [6]. Kawamura used conventional ultrasound, CDE, and enhanced CT to study the migratory spleen and found that the production of the migratory spleen is mostly due to congenital dysplasia or the relaxation of the splenic suspensory ligament, which leads to torsion of the spleen [7]. Sato is based on acoustic radiation force pulse imaging, and by using the working mechanism of acoustic pulse radiation force imaging and shear wave propagation, without manual pressure application, it provides the possibility of analyzing deep tissue compliance [8]. George proposed that contrast-enhanced ultrasound technology can dynamically observe the whole process of tumor blood perfusion, has a high ability to display small blood vessels, and has a high accuracy rate for kidney tumors [9].

This article uses transabdominal two-dimensional ultrasound to observe the changes of shear wave velocity in patients with chronic kidney disease in different stages and explores the application value of elastography technology in chronic kidney disease and further explores three-dimensional ultrasound kidney volume, elastography, and correlation of renal artery resistance index at different stages of chronic renal disease and its application value in the diagnosis of chronic renal disease, so as to provide timely clinical imaging report for early detection and early secondary preventive measures.

## 2. Diagnosis of Chronic Kidney Disease by Three-Dimensional Contrast-Enhanced Ultrasound Combined with Augmented Reality Medical Technology

### 2.1. Imaging Study of Chronic Kidney Disease

#### 2.1.1. Causes of Chronic Kidney Disease

Chronic kidney disease caused by diabetes and hypertension has a significant growth trend [10]. The occurrence and development of chronic kidney disease often shows a slow trend, which is easy to be ignored by people in the early stage of onset, and is often ignored in the course of disease development. Eventually, it missed the best time to treat chronic kidney disease [11, 12]. There are many factors that can cause people to develop chronic kidney disease. Common are age, high blood pressure, diabetes, and some patients using nephrotoxic drugs [8]. People with a family history of chronic kidney disease are also more likely to develop chronic kidney disease. And some people with obesity-metabolic syndrome and infectious diseases are also susceptible to chronic kidney disease [13, 14].

#### 2.1.2. Film Degree Exam

With the rapid development of imaging technology, researchers and physicians can obtain more useful imaging information through a variety of technical methods and in-depth morphological information exploration to provide clinical information on renal function.

*(1) Renal Radionuclide Imaging*. Since the resolution of renal nuclide manifestation is lower than that of other examinations, it cannot provide clear renal vascular images in clinical operations, nor can it provide clinical operations with the structure and relationship of kidney tissue and its surrounding tissues. The patient also needs other tests [15, 16].

*(2) Computed Tomography*. There are many researches on renal function, some of which can express the function of the kidney with specific values. CT perfusion scan has its unique role in this aspect. It has gradually begun to be applied to the research of quantitative analysis of renal function, affecting its accuracy, and leading to measurement errors [17, 18], and due to the necessary continuous perfusion parameters, the radiation dose that the patient needs to receive will greatly increase, which limits its clinical application to a greater extent.

*(3) Magnetic Resonance*. Magnetic resonance imaging is a non-invasive imaging examination method. Magnetic resonance can clearly and accurately display the changes in renal function, and it can also provide information on the anatomy of the kidney [19, 20]. There are many techniques for evaluating kidney function. Magnetic resonance is a new technique. It can not only show the changes of the kidney in morphology, but also give us more functional information of the kidney and the resolution of the magnetic resonance is high [21]. There is no need for a contrast agent, no radiation damage, no trauma.

#### 2.1.3. Ultrasound

Ultrasound diagnosis is widely used in clinics. It can not only clearly display the shape and structure of the kidney, but also dynamically observe its blood flow in real time [22], thereby reducing unnecessary invasive examinations and reducing damage to patients. And it can monitor patients in real time and evaluate the prognosis [23, 24].

*(1) Two-Dimensional Ultrasound*. Two-dimensional ultrasound is widely used in ultrasound inspection, and its impact is the greatest. When the human body's various layers of interfaces and tissue structures are passed through by the sound beam of two-dimensional ultrasound, the images it receives are captured according to the intensity of the light and shadow response. These images are composed of many points and arranged in order [25]. In real-time imaging in the examination of chronic kidney disease, two-dimensional ultrasound can regularly detect the various stages of chronic kidney disease. With the continuous development of chronic kidney disease, the kidney gradually becomes smaller, the cortex gradually becomes thinner, and the parenchymal echo is enhanced [26].

*(2) Color Doppler*. With the constant updating of medical technology, medical diseases are constantly improving. More and more hospitals are adopting color doppler ultrasound technology. This technology has become an important inspection method, combining doppler with ultrasound technology. The combination is doppler color ultrasound technology. Doppler ultrasound is an ultrasound that reflects the changing frequency of the body. Stereo and charts can show the frequency shift it produces [27, 28].

*(3) Elastography*. Acoustic radiation force pulse imaging is a kind of elastic imaging that is more suitable for kidney tissue. Therefore, it is a brand-new technology for detecting and evaluating the elasticity of kidney tissue. It is an elastic image produced without external force acting on deep tissue. If the tissue shows the same echo in the traditional ultrasound image, the acoustic radiation force pulse imaging is to obtain a quantitative elasticity value by compressing the sound wave energy to distinguish the softness and hardness of the deep tissue [29].

*(4) Three-Dimensional Ultrasound*. The vascular tree in the kidney can be reconstructed with color imaging of vascular energy and displayed in the form of spatial three-dimensional images, so as to show the shape, number, and distribution of blood vessels in the kidney. 3D ultrasound volume measurement technology can display multiple levels to display three mutually perpendicular planes that are not in the same plane at the same time. By arbitrarily paralleling and rotating these three planes, an ultrasound image with a stronger stereoscopic effect than two-dimensional ultrasound can be obtained [30], which can more intuitively reflect the morphology of the kidney and at the same time can collect more imaging information [31, 32].

### 2.2. Medical Image Enhancement Algorithm

#### 2.2.1. Histogram Equalization

In the original input image, the gray level with a relatively small number of pixels decreases and the gray level with a relatively large number of pixels expands [33]. This method can achieve the goal of improving the overall contrast of the image. The gray histogram of the image describes the relationship between the number of gray values in the input pixel and the relative frequency. The expression of the relationship is as follows:

(1) $$\begin{array}{c} p\left(r_{k}\right)=\frac{n_{k}}{n}. \end{array}$$

*r*_*k*_ in the formula is the *k* gray level of the image, and *n* is the total number of gray pixel values in the image. If we want to study the histogram balance algorithm in-depth, we first start with the introduction of the histogram equation under continuous conditions [34, 35] and build the following transformation:

(2) $$\begin{array}{c} s=T\left(r\right),\;0\leq r\leq 1. \end{array}$$

Formula (2) maps the gray value *r* in the input image to the new gray value *s*. In order to ensure that the grayscale and grayscale transformation sequence of the output image obtained after transformation remain the same as the original image, we know from probability theory

(3) $$\begin{array}{c} p_{s}\left(s\right)=p_{r}\left|\frac{dr}{ds}\right|, \end{array}$$

(4) $$\begin{array}{c} ds=p_{r}\left(r\right)dr. \end{array}$$

Then, integrate the two sides of equation (4) to get

(5) $$\begin{array}{c} s=T\left(r\right)=\int_{0}^{r}p_{r}\left(x\right)dx. \end{array}$$

Then, the probability density function of the *k* gray level is expressed as shown in equation (1). At this time, the transformation function of the histogram equalization is expressed as follows:

(6) $$\begin{array}{c} s_{k}=T\left(r_{k}\right)=\sum_{i=0}^{k}p_{r}\left(r_{i}\right)=\sum_{i=0}^{k}\frac{n_{i}}{n}\\ f\left(k\right)=f_{\min}+\left(f_{\max}-f_{\min}\right)\times s_{k}. \end{array}$$

Here, *f*_max_ is the maximum pixel value of the original image, *f*_min_ is the minimum pixel value of the original image, and *k* is the number of gray levels.

#### 2.2.2. Grayscale Transformation Method

The general expression of the grayscale transformation method is as follows:

(7) $$\begin{array}{c} g\left(x,y\right)=T\left[f\left(x,y\right)\right]. \end{array}$$

In the above formula, *f*(*x*, *y*) represents the input image, and *g*(*x*, *y*) represents the output image after grayscale transformation, and the grayscale transformation function is represented by *T*[].

*(1) Linear Grayscale Transformation*. If the original image is represented by *f*(*x*, *y*), and the grayscale range of the image is represented by [*m*, *n*], *g*(*x*, *y*) is the output image after grayscale transformation, and [*M*, *N*] is the grayscale range of the output image. At this time, the linear grayscale transformation expression is as follows:

(8) $$\begin{array}{c} g\left(x,y\right)=\frac{\left(N-M\right)\left[f\left(x,y\right)-m\right]}{n-m}+M,\\ g\left(x,y\right)=\left\{\begin{array}{cc} \frac{k_{1}}{a}, & 0\leq f\left(x,y\right)\leq a,\\ \frac{k_{2}-k_{1}}{b-a}\left[f\left(x,y\right)-a\right]+k_{1}, & a\leq f\left(x,y\right)\leq b,\\ \frac{L-1-k_{2}}{L-1-b}\left[f\left(x,y\right)-b\right]+k_{2}, & b\leq f\left(x,y\right)\leq L-1. \end{array}\right. \end{array}$$

The shape of the transformation function is controlled by point (*a*, *k*_1_) and point (*b*, *k*_2_). Only when *a* ≤ *b*, *k*_1_ ≤ *k*_2_ can the special and unique processing effect of piecewise linear function be shown [36, 37].

### 2.3. Nonlinear Gray Scale Transformation

Nonlinear transformation is developed under the condition that linear transformation cannot meet our requirements for processing images. The formula is as follows:

(9) $$\begin{array}{c} g\left(x,y\right)=e^{k\left[f\left(x,y\right)-b\right]}-1. \end{array}$$

The general expression of logarithmic transformation is as follows:

(10) $$\begin{array}{c} g\left(x,y\right)=C\times \;\log\left[l+f\left(x,y\right)-\min\right]. \end{array}$$

The overall effect of the medical image after logarithmic conversion is blurred. This is because the darkest area of the image is mapped to the brightest area, and the brightest area in the image is mapped to the darkest area, so the overall contrast of the image is lower and the grayscale is smaller.

#### 2.3.1. Image Sharpening Enhancement

*(1) Gradient Operator*. If *f*(*x*, *y*) is the original image, then the gradient value definition formula of *f*(*x*, *y*) at point (*x*, *y*) is expressed as follows:

(11) $$\begin{array}{c} G\left[f\left(x,y\right)\right]=\left[\begin{array}{c} \frac{\partial f}{\partial x}\\ \frac{\partial f}{\partial y} \end{array}\right]. \end{array}$$

The expression of the magnitude of the gradient is as follows:

(12) $$\begin{array}{c} \left|G\left[f\left(x,y\right)\right]\right|=\sqrt{{\left(\frac{\partial f}{\partial x}\right)}^{2}+{\left(\frac{\partial f}{\partial y}\right)}^{2}}. \end{array}$$

Most of the current medical images are digital images, so we have to consider how to solve the image gradient in the discrete case. Generally speaking, it is usually used to approximate the expression (11) with the search operation, as shown below:

(13) $$\begin{array}{c} \left|G\left[f\left(x,y\right)\right]\right|={\left\{{\left[f\left(x,y\right)-f\left(x+1,y\right)\right]}^{2}+{\left[f\left(x,y\right)-f\left(x,y+1\right)\right]}^{2}\right\}}^{1/2},\\ \left|G\left[f\left(x,y\right)\right]\right|\approx \left|f\left(x,y\right)-f\left(x+1,y\right)\right|+\left|f\left(x,y\right)-f\left(x,y+1\right)\right|. \end{array}$$

The size of the grayscale is proportional to the difference between the grayscale values of adjacent pixels in the two directions. Experiments show that the tilt value of the smooth area of the image is small, while the tilt value of the edge area of the image is higher. Using this, we can roughly distinguish the smooth and detailed areas of the image and then sharpen the edges of the details for the enhanced detail areas [35, 36]. The pixel value of the original image can be replaced with these calculated gradient values of each point to obtain a new gray value and a new output image. The formula is as follows:

(14) $$\begin{array}{c} g\left(x,y\right)=G\left[f\left(x,y\right)\right],\\ g\left(x,y\right)=\left\{\begin{array}{cc} G\left[f\left(x,y\right)\right], & G\left[f\left(x,y\right)\right]\geq T\\ f\left(x,y\right), & \left[f\left(x,y\right)\right]<T \end{array}\right., \end{array}$$

*T* represents the set threshold. When the gradient value of a certain area in the image is greater than the threshold, the pixel gray value of the original image is replaced with the gradient value; and when the gradient value of a certain area is less than this threshold, the original image the gray value does not change.

*(2) Laplacian*. *f*(*x*, *y*) represents the image to be enhanced, and the Laplacian differential definition of *f*(*x*, *y*) at point (*x*, *y*) is expressed as follows:

(15) $$\begin{array}{c} \nabla^{2}\left(x,y\right)=\frac{\partial^{2}f}{\partial x^{2}}+\frac{\partial^{2}f}{\partial y^{2}}. \end{array}$$

The general expression for enhancement using Laplace is as follows:

(16) $$\begin{array}{c} g\left(x,y\right)=f\left(x,y\right)-A\cdot \nabla^{2}f\left(x,y\right),\\ \nabla^{2}f\left(x,y\right)=\left[f\left(x+1,y\right)+f\left(x-1,y\right)+f\left(x,y+1\right)+f\left(x,y-1\right)\right]-4f\left(x,y\right). \end{array}$$

Since the second-order Laplacian operator can detect a line segment and a single point in an image, even when the image is affected by noise [38], even if the bright spot in the dark area becomes brighter, the algorithm will make the noise have more influence. Therefore, the noise algorithm of the algorithm must be taken into account when using the Laplace operator.

## 3. Experimental Design for Diagnosis of Chronic Kidney Disease

### 3.1. Test Subject

The subjects of this experimental study are patients with chronic kidney disease hospitalized in the department of nephrology of X Hospital from June 2019 to June 2020, including 160 males and 140 females, all of whom were diagnosed as chronic kidney disease by clinical or renal pathological biopsy, and all meet the K/DOQI diagnostic criteria for chronic kidney disease. All selected subjects meet the criteria. They are between 20 and 75 years old and have a BMI of 18.5–23.9 kg/m^2^. Diabetic nephropathy, diabetic nephropathy, and diabetic nephropathy can be ruled out by consulting medical records. The test subjects were patients with diabetic nephropathy, hypertensive nephropathy, renal artery stenosis, acute heart failure, and hepatorenal syndrome. The 300 patients were divided into 5 groups according to their pathological stages, with 60 patients in each group, to explore the correlation of properties such as three-dimensional ultrasound kidney volume in different stages of chronic kidney disease. The research project was approved by the hospital ethics committee, and all subjects had informed consent.

### 3.2. Instruments and Methods

#### 3.2.1. Instruments

The SIEMENS ACUSON S2000 color doppler ultrasound system produced by Siemens was equipped with a VTQ quantitative analysis system and a 4C1 abdominal probe; the Philips iu Elite color doppler ultrasound system produced by Philips was equipped with an X6−1 abdominal probe, configured C5−1 abdominal probe.

#### 3.2.2. Methods

Before the examination, the general information of all the examinees was registered, including age, height, weight, etc., and relevant information was entered in combination with medical records. And the subject was instructed to fast for at least 8 hours before the examination and empty his bowels. After the examinee was ready, he was asked to lie on his side on the examination table. First the C5−1 abdominal probe of the PHILIPS iu Elite instrument was used to perform routine two-dimensional ultrasound examination to observe the structure and size of the kidney, cortical thickness, internal echo, etc., and then color doppler was used to observe the blood flow of the renal artery, the color doppler sampling volume was placed in the renal artery, and then the subject was asked to hold his breath. Once there was a clearer arterial blood flow range, resistance index was measured by detection method and the value of renal artery resistance index was recorded. Each item was counted 5 times and then the mean value was taken as the survey item.

### 3.3. Observation Index

Chronic kidney disease is divided into early stage and late stage. Among them, chronic kidney disease stage 1, chronic kidney disease stage 2, and chronic kidney disease stage 3 are the early stage, and the chronic kidney disease stage 4 and chronic kidney disease stage 5 are the advanced stage. Based on this, we study the change of the area under the renal artery resistance index curve. Then, the area under the curve for the diagnosis of early- and late-stage chronic kidney disease is calculated by using the receiver operating characteristic curve to calculate the elasticity value, three-dimensional volume, and renal artery resistance index.

### 3.4. Statistical Data Processing Method

SPSS23.0 software was used for data processing, and count data was expressed as percentage (%), *k* is the number of data in this experiment, *σ*^2^ is the variance of all survey results, and *P* < 0.05 indicates that the difference is statistically significant. The formula for calculating reliability is shown in equation (16).

(17) $$\begin{array}{c} a=\frac{k}{k-1}\left(1-\frac{{\sum \sigma_{i}}^{2}}{\sigma^{2}}\right). \end{array}$$

## 4. Experimental Diagnosis of Chronic Kidney Disease

### 4.1. Evaluation Index System Based on Index Reliability Testing

It is generally believed that the *α* coefficient above 0.8 indicates that the effect of the index setting is very good, and above 0.7 is also acceptable. Here, we analyze the reliability of each type of object, and the reliability index we choose for each type of object is slightly different. The results are shown in Table 1. In the experimental stage, our experimental object is the artistic visual form of ceramic murals and the data source is the questionnaire that was issued and retrieved. Here, we publish questionnaires by age group to reduce significant differences.

It can be seen from Figure 1 that the data obtained from various indicators such as elasticity value, three-dimensional volume, and renal artery resistance index have a very good effect on this experiment (*α* > 0.8). The data obtained from the correlation between the arterial resistances index have an acceptable impact on this experiment (*α* > 0.7). The three-dimensional ultrasound combined with augmented reality medical technology is very necessary for the diagnosis of chronic kidney disease.

### 4.2. Analysis Based on the Patient's Elastic Value, Three-Dimensional Volume, and Renal Artery Resistance Index

#### 4.2.1. Analysis Based on the Patient's Elasticity Value

One day after ultrasound detection, ultrasound-guided puncture biopsy was performed on the left lower pole of the patient's renal parenchyma. The change in renal arterial transparency refers to renal hyalinosis. Here, the collected data of the patient's renal parenchymal elasticity are analyzed, and the results are shown in Table 2.

In chronic kidney disease subjects, the comparison results of renal parenchymal elasticity values among multiple groups are shown in Figure 2. As the stage of chronic kidney disease increases, the renal parenchymal elasticity values decrease, *P* < 0.05; the difference is statistically significant, indicating that the value of renal parenchymal elasticity is negatively correlated with the stage of chronic kidney disease; that is to say, the quantitative analysis of tissue by acoustic palpation detects that the value of renal parenchymal elasticity decreases as the stage of chronic kidney disease increases.

#### 4.2.2. Analysis Based on the Patient's Three-Dimensional Volume

One day after ultrasound detection, ultrasound-guided puncture biopsy was performed on the left lower pole of the patient's renal parenchyma to measure the size of the kidney in different stages of the same patient. Here, the data collected from the three-dimensional volume of the patient's renal parenchyma were analyzed. The results are as shown in Table 3.

In chronic kidney disease subjects, the comparison of the three-dimensional renal parenchymal volume among multiple groups is shown in Figure 3. As the stage of chronic kidney disease increases, the three-dimensional renal parenchymal volume decreases, *P* < 0.05; the difference is statistically significant, indicating that the three-dimensional volume of the renal parenchyma is also negatively correlated with the stage of chronic kidney disease; that is to say, the three-dimensional volume of the renal parenchyma decreases as the stage of chronic kidney disease increases.

#### 4.2.3. Analysis Based on the Patient's Renal Artery Resistance Index

One day after ultrasound detection, ultrasound-guided puncture biopsy was performed on the left lower pole of the patient's renal parenchyma. The progressive decline in renal function is characterized by the destruction of microvascular structures and the accumulation of fibrotic matrix. Here, the data were collected for the patient's renal artery resistance index and the analysis was performed and the results are shown in Table 4.

In chronic kidney disease subjects, the comparison results of the renal artery resistance index among multiple groups are shown in Figure 4. As the stage of chronic kidney disease increases, the renal artery resistance index value becomes larger, *P* < 0.05; the difference is the statistical significance that shows that the renal artery resistance index is positively correlated with the stage of chronic renal disease, which means that the renal artery resistance index increases with the increase of the chronic renal disease stage.

### 4.3. Analysis Based on the Correlation between the Patient's Elastic Value, Three-Dimensional Volume, and Renal Artery Resistance Index

#### 4.3.1. Analysis Based on the Correlation between the Patient's Elasticity Value and the Renal Artery Resistance Index

One day after the ultrasound detection, ultrasound-guided puncture biopsy was performed on the left lower pole of the patient's renal parenchyma. Here, the relationship between the patient's elasticity value and the renal artery resistance index was analyzed, and the results are shown in Table 5.

With the increase in the stages of chronic kidney disease, there is a certain correlation between the elasticity value and the renal artery resistance index in the parameters of the ultrasound examination, as shown in Figure 5. Pearson correlation analysis can be used to conclude that the smaller the elasticity value, the larger the arterial resistance index, which means that the elasticity value and the renal artery resistance index are negatively correlated with the increase of the stage of chronic kidney disease, *P* < 0.05, which is statistically significant.

#### 4.3.2. Analysis Based on the Correlation between the Patient's Renal Artery Resistance Index and Volume

One day after ultrasound detection, ultrasound-guided puncture biopsy was performed on the left lower pole of the patient's renal parenchyma. Here, the relationship between the patient's renal artery resistance index and volume was analyzed, and the results are shown in Table 6.

As the stages of chronic kidney disease increase, there is also a certain correlation between the renal artery resistance index and volume, as shown in Figure 6. Using Pearson correlation analysis, it can be concluded that the smaller the renal artery resistance index, the larger the volume. It shows that the renal artery resistance index and volume are negatively correlated with the increase of chronic kidney disease stages, *P* < 0.05, which is statistically significant.

#### 4.3.3. Analysis Based on the Correlation between the Patient's Elasticity and Volume

One day after the ultrasound detection, ultrasound-guided puncture biopsy was performed on the left lower pole of the patient's renal parenchyma. Here, the relationship between the patient's elasticity and volume was analyzed, and the results are shown in Table 7.

As the stages of chronic kidney disease increase, there is also a significant correlation between elasticity and volume, as shown in Figure 7. According to Figure 7, elasticity and volume showed a significant positive correlation (*P* < 0.05), with the increase in the stage of chronic kidney disease, which shows that it is statistically significant.

## 5. Conclusions

Transabdominal two-dimensional ultrasound elastography ultrasound technology can be used to observe the shear wave velocity of the renal cortex of patients with chronic kidney disease. It is not only easy to operate, but also reproducible, and can provide a new imaging examination for patients with chronic kidney disease. Basis: trans-abdominal three-dimensional ultrasound examination technology can more intuitively observe the shape, structure, volume, etc. of the kidney in patients with chronic kidney disease, and its reproducibility is good, which can provide patients with a more intuitive imaging examination method, and at the same time for chronic kidney disease the patient provides a new noninvasive inspection method. As the stages of chronic kidney disease increase, the three-dimensional volume of the kidney shows a decreasing trend, the renal artery resistance index shows an increasing trend, and the shear wave velocity shows a decreasing trend, and there is a certain correlation between the three.

Three-dimensional contrast-enhanced ultrasound is a commonly used clinical imaging method for renal tumors. It is generally accepted by patients and clinicians. It mainly observes the enhancement degree, enhancement mode, renal vein, and inferior vena cava for tumor thrombus and lymph node the metastasis and the invasion of tissues around the kidney can make a more accurate qualitative diagnosis and staging diagnosis of renal lesions. As the most advanced ultrasound examination technology, contrast-enhanced ultrasound makes up for the deficiencies of conventional ultrasound and color ultrasound. It has unique advantages such as no radiation, low allergy, strong adaptability, and no nephrotoxicity, and can dynamically observe the blood perfusion of the tumor. The whole process has been rapidly developed and widely used in clinical practice in recent years, providing a new clinical examination method.

Through three-dimensional imaging to measure the volume, we confirmed that the kidney volume of patients with severely damaged kidneys was significantly reduced, while in patients with mildly damaged kidneys, the volume change has no significant statistical significance, thus confirming that three-dimensional volume imaging can only be used to reflect the kidneys. It is an indicator of severely impaired function and cannot be used as an indicator of early renal impairment. In this paper, the sampling depth of kidney elasticity is adjusted to reduce the influence of elasticity depth on the elasticity value, which greatly increases the reliability of the results of this study. Ultrasound imaging can perform early screening of asymptomatic patients, which is conducive to early clinical detection of chronic kidney disease, early symptomatic intervention measures, and monitoring of the occurrence and development of the disease to prevent it from developing into end-stage renal failure, and kidney replacement is needed for life treatment.

## Figures and Tables

**Figure 1:** Indicator reliability test analysis chart.

**Figure 2:** Comparison analysis chart of VTQ value between groups.

**Figure 3:** Three-dimensional volume comparison between groups.

**Figure 4:** Ramsay sedation score analysis diagram at each moment during anesthesia.

**Figure 5:** Correlation analysis chart between elasticity value and renal artery resistance index.

**Figure 6:** Analysis chart of the correlation between renal artery resistance index and volume.

**Figure 7:** Correlation analysis graph between elasticity value and volume.

**Table 1:** Data sheet of evaluation index system for index reliability testing.

	Very clear	Clear	General	Not clear	Chaotic	Alpha
Elasticity	0.305	0.337	0.183	0.096	0.079	0.9133
Three-dimensional volume	0.249	0.287	0.216	0.162	0.086	0.8196
Renal artery resistance index	0.217	0.241	0.297	0.187	0.058	0.8362
Elasticity and renal artery resistance index	0.112	0.186	0.352	0.197	0.153	0.7335
Renal artery resistance index and volume	0.146	0.172	0.398	0.203	0.081	0.7829
Elasticity and volume	0.204	0.162	0.313	0.173	0.148	0.7713

**Table 2:** Data table for comparison of VTQ values between groups.

CKD staging	Glomerular hyperplasia	Segmental glomerular damage	Glomerulosclerosis	Renal interstitial fibrosis	Renal tubule atrophy	*P*
CKD1 period	2.78	2.91	2.74	2.91	2.63	<0.001
CKD2 period	2.28	2.43	2.47	2.34	2.33	<0.001
CKD3 period	1.92	1.95	1.86	1.93	1.97	<0.001
CKD4 period	1.34	1.13	1.03	1.21	1.12	<0.001
CKD5 period	0.66	0.80	0.63	0.59	0.79	<0.001

**Table 3:** Three-dimensional volume comparison data table.

CKD staging	Three-dimensional volume	Kidney length	Renal parenchymal thickness	Cortical thickness	Medulla area	*P*
CKD1 period	2.38	2.89	2.40	2.81	2.75	<0.001
CKD2 period	1.90	2.26	2.19	2.32	2.04	<0.001
CKD3 period	1.52	1.83	1.64	1.39	1.53	<0.001
CKD4 period	1.67	1.32	1.02	1.40	1.50	<0.001
CKD5 period	1.09	1.00	0.98	0.92	1.19	<0.001

**Table 4:** Ramsay sedation score data sheet at each moment during anesthesia.

CKD staging	Arterial resistance index	Arterial acceleration time	Arterial resistance sensitivity	Arterial resistance specificity	Arterial resistance accuracy	*P*
CKD1 period	0.59	0.56	1.15	0.97	1.02	<0.001
CKD2 period	1.04	1.73	1.71	1.14	1.27	<0.001
CKD3 period	1.67	1.94	1.56	1.92	1.53	<0.001
CKD4 period	2.06	2.29	2.30	2.04	1.96	<0.001
CKD5 period	2.94	2.82	2.40	2.67	2.69	<0.001

**Table 5:** Correlation data table between elasticity value and renal artery resistance index.

CKD staging	0.5 h	1 h	2 h	4 h	8 h	12 h	*P*
CKD1 period	2.77	2.54	2.80	2.38	2.82	2.73	0.001
CKD2 period	2.41	2.07	2.15	2.05	2.45	2.08	0.002
CKD3 period	1.69	1.69	1.90	1.43	1.65	1.71	0.004
CKD4 period	1.42	1.51	1.42	1.44	1.21	1.35	0.005
CKD5 period	0.74	0.84	1.16	0.90	0.89	1.04	0.008

**Table 6:** Correlation data table between renal artery resistance index and volume.

CKD staging	0.5 h	1 h	2 h	4 h	8 h	12 h	*P*
CKD1 period	2.70	2.49	2.78	2.67	2.54	2.65	0.001
CKD2 period	2.18	2.09	2.45	2.43	2.05	2.45	0.002
CKD3 period	1.85	1.75	2.14	1.80	1.87	2.13	0.004
CKD4 period	1.42	1.55	1.21	1.71	1.24	1.25	0.005
CKD5 period	1.09	1.21	1.21	1.31	1.01	1.29	0.008

**Table 7:** Correlation data table between elasticity value and volume.

CKD staging	0.5 h	1 h	2 h	4 h	8 h	12 h	*P*
CKD1 period	1.03	1.02	1.15	1.25	0.80	1.22	0.001
CKD2 period	1.33	1.23	1.54	1.37	1.77	1.21	0.002
CKD3 period	1.74	1.84	1.56	1.71	1.77	1.77	0.004
CKD4 period	2.35	2.30	2.22	2.27	1.88	2.26	0.005
CKD5 period	2.36	2.48	2.90	2.59	2.80	2.68	0.008

## Data Availability

No data were used to support this study.
